The article "Effects of Aerosol Inhalation Combined with Intravenous Drip of Polymyxin B on Bacterial Clearance, Symptoms Improvement, and Serum Infection Indexes in Patients with Pneumonia Induced by Multidrug-Resistant Gram-Negative Bacteria" was published in 2022. Journal: Emerg Med Int.

# Effects of Aerosol Inhalation Combined with Intravenous Drip of Polymyxin B on Bacterial Clearance, Symptoms Improvement, and Serum Infection Indexes in Patients with Pneumonia Induced by Multidrug-Resistant Gram-Negative Bacteria

**DOI:** 10.1155/2022/5244538

**Published:** 2022-08-28

**Authors:** Hanlu Lin, Xiaobo Liu, Pengfei Sun

**Affiliations:** Department of Pharmacy, Hospital of Chengdu University of Traditional Chinese Medicine, Chendu, Sichuan 610032, China

## Abstract

In recent years, the incidence of pneumonia caused by multidrug-resistant (MDR) Gram-negative bacteria (*G*−) has increased year by year. Polymyxin B has a good clinical effect in the treatment of MDR, but there is controversy about the administration route of this drug. In this study, we retrospectively analyzed the clinical data of 84 cases of MDR Gram-negative bacterial pneumonia, and aimed to explore the effects of aerosol inhalation combined with intravenous polymyxin B infusion on the bacterial clearance, symptom improvement, and serum infection indexes of MDR patients on the patients with Gram-negative (*G*−) bacterial pneumonia. The results show that aerosol inhalation combined with intravenous drip of polymyxin B can improve bacterial clearance rate, reduce levels of serum inflammatory factors, and improve clinical symptoms in patients with pneumonia induced by MDR G-bacteria.

## 1. Introduction

In recent years, with the widespread use of broad-spectrum antibiotics, the incidence of pneumonia caused by multidrug-resistant (MDR) Gram-negative (*G*−) bacteria is increasing year by year, which has brought greater difficulties and challenges to the clinical anti-infection treatment [1, 2]. Polymyxin B is one of the peptide antibacterial drugs in clinical practice. It was widely used in the treatment of patients with Gram-negative bacilli in the 1960s, but it was gradually abandoned in clinic because of many adverse reactions. However, with the increasing incidence of MDR in recent years, the role of traditional antibacterial drugs has been limited [3]. Polymyxin B has been reused in the clinical treatment of MDR due to its good antibacterial activity [4]. Foreign studies have found that polymyxin B has a good clinical therapeutic effect in the treatment of MDR, but the route of administration of the drug is controversial. Intravenous administration is a common route of administration, which can significantly improve the clinical symptoms of patients [5]. Other scholar have reported that aerosol inhalation therapy can make polymyxin B enter the airway of patients in the form of aerosol to play a full anti-inflammatory role, and has the advantages of rapid onset, and can rapidly reduce the level of serological infection [4]. However, due to the lack of uniform clinical reports on the drug regimen of polymyxin B in patients with pneumonia caused by MDR Gram-negative (*G*−) bacteria, this study was designed to investigate the effects of aerosol inhalation combined with intravenous polymyxin B infusion on bacterial clearance, symptom improvement, and serum infection index of patients with multiresistant Gram-negative bacterial pneumonia.

## 2. Materials and Methods

### 2.1. General Information

A total of 84 patients with pneumonia caused by MDR Gram-negative (*G*−) bacteria who were admitted to the intensive care center of our hospital from January 2020 to January 2022 were retrospectively selected as the research subjects. According to the different administration methods of polymyxin B, 40 patients who were treated by intravenous drip alone from January 2020 to January 2021 were included in the control group. Forty-four patients who received intravenous drip combined with aerosol inhalation therapy according to the international guidelines for optimal application of prime factors were included in the observation group.

### 2.2. Inclusion Criteria

(1) In line with the Chinese Medical Association's guidelines for the diagnosis of pneumonia [6]; (2) MDR Gram-negative (*G*−) bacteria detected by sputum culture, and sensitive to polymyxin B; (3) the treatment time of the two groups was ≥3d.

### 2.3. Exclusion Criteria

(1) Simultaneous infection with multiple MDR Gram-negative (*G*−) pathogens; (2) severe liver and kidney insufficiency; (3) combined with malignant tumors and incomplete clinical data.

### 2.4. Treatment Options

Both groups received routine broad-spectrum antibiotics for anti-infection, phlegm reduction, nutrition, and electrolyte supplementation.

The control group was treated with simple intravenous drip of polymyxin B for the treatment of pneumonia caused by MDR Gram-negative (*G*−) bacteria. The first dose was 2.0 mg/kg, and the adjusted dose was 1.25 mg/kg on the 2nd day, once every 12 hours, twice a day.

According to the recommendation of the international consensus guideline [4] for the optimal application of polymyxins, the observation group used the regimen of intravenous drip combined with aerosol inhalation to treat pneumonia caused by MDR Gram-negative (*G*−) bacteria. 25 mg/kg nebulized inhalation therapy twice a day.

### 2.5. Observation Indicators

1. Judgment of curative effect: after the course of polymyxin B treatment, the bacterial clearance rate and clinical efficacy of patients with pneumonia caused by MDR Gram-negative (*G*−) bacteria were evaluated with reference to the Technical Guidelines for Clinical Trials of Antibacterial Drugs [7]. During the treatment process, the sputum culture was sent for inspection on the 3rd, 7th, and 14th days, respectively, to understand the microbial clearance. ① Cleared: 3 consecutive sputum culture results showed negative; replacement: 3 consecutive sputum cultures result in the disappearance of the pathogenic bacteria, but the growth of other pathogens; ② not cleared: sputum culture results in the original pathogen infection. The total bacterial clearance = clearance + replacement.
2. Clinical efficacy: ① markedly effective means that the condition has improved significantly, and one of the pathogenic bacteria culture, laboratory indicators and clinical signs has not returned to normal; ② effective means that the condition has improved, but the pathogenic bacteria culture, laboratory indicators and clinical signs are not significantly improved; ③ invalid means that the condition has not improved or even worsened. The total effective rate = markedly effective + effective rate.
3. Clinical symptoms: the time for body temperature to return to normal, time for disappearance of rales, time for leukocyte recovery, and X-ray recovery time were observed and recorded in the two groups.
4. Infection indexes: before treatment, 3 days after treatment, and 7 days after treatment, 3–5 ml fasting venous blood was collected from patients, centrifuged (3 500 rpm, 10 min), the supernatant was separated, and lipopolysaccharide (LPS) and interleukin 6 were detected by ELISA. IL-6, C-reactive protein (CRP), and procalcitonin (PCT) levels, strictly follow the instructions of the kit (Shanghai Guduo Biotechnology Co., Ltd.).
5. Incidence of nephrotoxic reaction: the number of nephrotoxic reactions occurred in the two groups of patients during treatment were observed and recorded.

### 2.6. Statistical Processing

The SPSS 21.0 software was used to organize and analyze the clinical data of patients with pneumonia caused by MDR Gram-negative (*G*−) bacteria included in this study. The measurement data that meet the normal distribution are expressed as the mean ± standard deviation ($\bar{x}$ ± *S*). Differences between the two groups were compared using *t*-test analysis. The count data are all expressed as rate (%), and comparisons between categorical data were performed using the *χ*^2^ test. Differences were considered statistically significant at *P* < 0.05.

## 3. Results

### 3.1. General Data

There were no significant differences in gender, age, acute physiology, chronic health score II (APACHE II), and distribution of pathogenic bacteria and underlying diseases between the two groups (*P* > 0.05), as shown in Table 1.

### 3.2. Comparison of Clinical Efficacy between the Two Groups of Patients

After treatment, the total effective rate of the observation group was 95.45%, which was significantly higher than that of the control group, 80.00% (*P* < 0.05), as shown in Table 2.

### 3.3. Comparison of Bacterial Clearance Rates between the Two Groups of Patients

After the sputum culture test on the 3rd, 7th, and 14th days after treatment, a total of 71 pathogenic bacteria were detected in 44 patients in the observation group, 64 were eliminated and 4 were replaced (2 *Pseudomonas aeruginosa* were replaced by *Escherichia coli*, and 2 strains of *Acinetobacter baumannii* were replaced by *Pseudomonas aeruginosa*), 3 strains were not cleared (2 strains of *Acinetobacter baumannii* and 1 strain of *Staphylococcus aureus*), and the total clearance rate was 90.14%. A total of 67 pathogenic bacteria were detected in 40 patients in the control group, 52 were eliminated, and 10 were replaced (6 *Pseudomonas aeruginosa* were replaced by *Acinetobacter baumannii*, 4 *Staphylococcus aureus* were replaced by *Pseudomonas aeruginosa*), 5 strains were not cleared (3 strains of *Escherichia coli* and 2 strains of *Pseudomonas aeruginosa*), the total clearance rate was 77.61%, and the total clearance rate of the observation group was significantly lower than that of the control group (*P* < 0.05), as shown in Table 3.

### 3.4. Comparison of Clinical Symptoms Improvement between Two Groups of Patients

The time for body temperature to return to normal, the time for disappearing rales, the time for leukocyte recovery and the time for X-ray recovery in the observation group were all shorter than those in the control group (*P* < 0.05), as shown in Table 4.

### 3.5. Comparison of Serum Infection Indicators between the Two Groups of Patients

Before treatment, there was no significant difference in serum LPS, IL-6, CRP, and PCT levels between the two groups (*P* > 0.05). Compared with before treatment, it showed a gradual downward trend (*P* < 0.05), and the downward trend in the observation group was more obvious. There was no significant difference in serum LPS, IL-6, CRP, and PCT levels between the two groups 14 days after treatment (*P* > 0.05), as shown in Figure 1.

### 3.6. Comparison of the Incidence of Nephrotoxic Reaction between the Two Groups of Patients

During the treatment period, the number of nephrotoxicity cases in the observation group was 3 cases (6.82%), and there was no significant difference compared with 4 cases (10.00%) in the control group (*P* > 0.05).

## 4. Discussions

Although the aseptic awareness of medical staff has been continuously enhanced and the isolation protection system of patients has been continuously improved, the incidence of MDR is still relatively high, which directly cause hospitalization of patients. Prolonged time and increased hospitalization costs lead to a waste of medical resources [8, 9]. The pathogenic bacteria mainly include *Klebsiella pneumoniae* and *Pseudomonas aeruginosa*. Polymyxin B is sensitive to many of these pathogens, and it has a good effect in clinical treatment.

Controlling bacterial infection and killing the activity of pathogenic bacteria are the principles of medication for the treatment of MDR Gram-negative (*G*−) bacterial pneumonia [10]. The results of this study showed that after treatment, the total bacterial clearance rate of the observation group was 90.14%, which was significantly higher than that of the control group, which was 77.61%, and the time for body temperature to return to normal, the time for disappearing rales, the time for leukocyte recovery, and the time for X-ray recovery in the observation group were shorter than the control group. It shows that aerosol inhalation combined with intravenous infusion of polymyxin B has a good bacterial clearance effect and improves the clinical symptoms of patients. The reason may be related to the pharmacological mechanism of polymyxin B [11, 12]. After the cationic lipopeptide in polymyxin B interacts with bacterial outer membrane lipopolysaccharide, it replaces the stable magnesium ions and calcium ions on the cell membrane, and increase the permeability of the cell membrane, resulting in disorder of the cell membrane structure, so that the intracellular substances in the bacteria are penetrated to crack and die, so it has a better bactericidal effect, and the combined treatment has a higher bacterial clearance rate [12].

This study found that after treatment, the total effective rate of the observation group was 95.45%, significantly higher than the control group's 80.00%. Analysis of the reasons shows that the molecular weight of polymyxin B is relatively large, and the amount of circulating into the alveoli after intravenous administration is relatively small. Combined with atomization treatment, the drug directly acts on the lesion site, which is beneficial to increase the penetration of antibiotics into the lower respiratory tract, so that the drug can reach a certain bactericidal concentration at the target, so the effect of drug treatment can be improved.

Pulmonary infection in patients with MDR Gram-negative (*G*−) bacteria pneumonia is a gradual process. LPS is the main component of the bacterial wall, which can participate in and activate inflammatory cytokines, thereby increasing the expression level of inflammatory factors. IL-6 is activated. Lymphokines produced by T cells and fibroblasts [13] have high expression levels when the body is infected. CRP is a protein that rises sharply in plasma when the body is infected or tissue damaged, which can activate complement and enhance the phagocytosis of phagocytes to play an opsonizing role. PCT can reflect the active degree of systemic inflammation in the body, and it is significantly increased in severe bacterial, fungal, and parasitic infections and sepsis [14, 15]. Pathogenic bacteria and airway secretions in patients with MDR Gram-negative (*G*−) pneumonia accumulate in the lungs, stimulate the production of mononuclear macrophages and neutrophils, and cause the body to secrete a large amount of IL-6, leading to systemic inflammatory response, and CRP and PCT were significantly increased. In this study, the levels of serum LPS, IL-6, CRP, and PCT in the two groups were gradually decreased at 3 d, 7 d, and 14 d after treatment compared with those before treatment, and the decrease trend was more obvious in the observation group. There was no significant difference in serum LPS, IL-6, CRP, and PCT levels between the two groups 14 days after treatment, suggesting that the two groups of treatment programs have good anti-infective effects. However, the results of this study showed that aerosol inhalation combined with intravenous infusion of polymyxin B can significantly reduce the level of serum inflammation, which mean that aerosol inhalation combined with polymyxin B intravenous infusion is effective in a short term and the anti-infection effect is more obvious.

During the treatment period, the number of nephrotoxicity cases in the observation group was 3 cases (6.82%), which was not significantly different from 4 cases (10.00%) in the control group. Many previous studies have reported [16, 17] that nephrotoxicity is the most common adverse reaction in the clinical application of polymyxin B. Combined with the conclusions of this study, some differences may be related to the relatively small number of samples included in this study. In the future, the expanded sample size and sample inclusion criteria will be discussed and studied in depth.

In conclusion, aerosol inhalation combined with intravenous infusion of polymyxin B can improve the bacterial clearance rate in patients with pneumonia caused by MDR Gram-negative (*G*−) bacteria, which is beneficial to improve clinical symptoms and reduce the level of serum inflammatory infection.

## Figures and Tables

**Figure 1:** Comparison of serum infection indicators between the two groups of patients.

**Table 1:** Comparison of general data of the two groups of patients (±*s*).

Group	Observation group (*n* = 44)	Control group (*n* = 40)	*t/χ * ^2^	*P* value
Gender			2.092	0.148
Male	29 (65.91)	32 (80.00)		
Female	15 (34.09)	8 (20.00)		

Age (year)	60.36 ± 2.98	60.77 ± 3.36		
APACHE II (score)	14.36 ± 2.28	14.98 ± 2.44	0.593	0.556

Pathogenic bacteria (strain)			0.672	0.955
*Pseudomonas aeruginosa*	20 (14.49)	21 (15.22)		
*Acinetobacter baumannii*	16 (11.59)	15 (10.87)		
*Escherichia coli*	17 (12.32)	14 (10.14)		
*Staphylococcus aureus*	12 (8.70)	13 (9.42)		
Other	6 (4.35)	4 (2.90)		

Combined hypertension			0.585	0.444
Yes	12 (27.27)	14 (35.00)		
No	32 (72.73)	26 (65.00)		

Combined coronary heart disease			1.006	0.316
Yes	10 (22.73)	13 (32.50)		
No	34 (77.27)	27 (67.50)		

**Table 2:** Comparison of clinical efficacy between the two groups of patients (*n*, %).

Group	Number of cases	Significant effect	Effective	Invalid	Total efficiency
Observation group	44	31 (70.45)	11 (25.00)	2 (4.55)	42 (95.45)
Control group	40	22 (55.00)	10 (25.00)	8 (20.00)	32 (80.00)
*χ * ^2^	—				4.772
*P* value	—				0.029

**Table 3:** Comparison of bacterial clearance rates between the two groups on the 3rd, 7th, and 14th days after treatment (*n*, %).

Group	*n*	3rd day after treatment	7th day after treatment	14th day after treatment
Observation group	71	39 (54.93)	45 (63.38)	64 (90.14)
Control group	67	34 (50.75)	42 (62.69)	52 (77.61)
*χ * ^2^	—	0.242	0.007	4.038
*P* value	—	0.623	0.933	0.044

**Table 4:** Comparison of clinical symptoms improvement between the two groups ($\bar{x}$ ± *S*).

Group	Number of cases	Temperature recovery time (d)	Rales disappearing time (d)	White blood cell recovery time (d)	X-ray recovery time (d)
Observation group	44	7.69 ± 1.26	10.34 ± 2.32	11.63 ± 2.56	10.93 ± 2.14
Control group	40	9.57 ± 0.99	12.53 ± 2.96	13.74 ± 2.98	12.68 ± 2.28
*χ * ^2^	—	7.603	3.774	3.481	3.627
*P* value	—	<0.001	<0.001	<0.001	<0.001

## Data Availability

The data can be obtained from the author upon reasonable request.
